# Application of Single-Hole Laparoscopy and Sentinel Lymph Node Imaging in Early Endometrial Carcinoma in Special Population

**DOI:** 10.1155/2021/9285708

**Published:** 2021-09-28

**Authors:** Jianqing Zhou, Weili Zhu, Tao Zhu, Xuedong Tang

**Affiliations:** ^1^Department of Gynecology, Jiaxing University Affiliated Women and Children Hospital, Jiaxing, Zhejiang 314000, China; ^2^Department of Gynecologic Oncology, Zhejiang Cancer Hospital, 38 Guangji Road, Hangzhou, Zhejiang 310022, China

## Abstract

**Aim:**

To explore the clinical efficacy of single-hole laparoscopy combined with sentinel lymph node imaging in the treatment of early endometrial carcinoma in a special population.

**Method:**

A retrospective analysis was made on the clinicopathological data of 8 patients with early endometrial carcinoma who underwent extra fascial total hysterectomy plus double adnexal resection and pelvic sentinel lymphadenectomy by transumbilical single-hole laparoscopy in Jiaxing Maternal and Child Health Hospital from Apr. 2019 to Apr. 2021.

**Result:**

Single-hole laparoscopy and sentinel lymph node imaging were successfully performed in 8 patients with early endometrial carcinoma, and none of them was converted to porous or laparotomy. At the same time, all 8 patients have a high demand for body shape. All FIGO pathological grades were grade I before operation. Operation time is 160.87 ± 40.61 min, amount of bleeding is 68.75 ± 12.31 ml, the catheter was removed for 2 days, anal exhaust time is 30.13 ± 10.99 h, and postoperative hospital stay is 4.00 ± 1.07 d. There was no related organ injury during the operation, no case of blood transfusion, or case of poor wound healing. The evaluation of postoperative satisfaction was very satisfactory.

**Conclusion:**

The application of single-hole laparoscopy and sentinel lymph node imaging in the treatment of early endometrial carcinoma in the special population should be safe and feasible with high satisfaction.

## 1. Introduction

In recent years, endometrial cancer shows a younger trend, and with the enhancement of people's awareness of disease and health, most endometrial cancers are found early. It brings new challenges to our gynecological oncologists for those special people, that is, those who have a high demand for their body shape, and the pursuit of accurate treatment and beauty is getting higher and higher. The gynecological oncology team of Jiaxing Maternal and Child Health Hospital used sentinel lymph node imaging technique to reduce the difficulty of operation for endometrial cancer and combined with single-hole laparoscopy to achieve minimally noninvasive, achieving a combination of precision and beauty. The treatments of 8 cases of early endometrial carcinoma are as follows:

## 2. Data Sources

The clinicopathological data of 8 patients with early endometrial carcinoma who underwent extra fascial total hysterectomy plus double adnexal hysterectomy and pelvic sentinel lymphadenectomy in the Department of Gynecology of Jiaxing Maternal and Child Health Hospital from Apr. 2019 to Apr. 2021 were collected. Patient age is 38-52 y. BMI (body mass index) is 22.39 ± 1.61, 20.4-24.3 kg/m^2^; there are 6 premenopausal women and 2 postmenopausal women. There was 1 yoga instructor, 1 dance trainer, 1 primary school English teacher, and 5 freelancers among the 8 patients with early endometrial cancer. And they all have high requirements for the appearance of the body. In these patients, one had a previous history of operation and 1 case of cesarean section (bikini incision). All 8 cases signed the informed consent form before the operation, which was discussed and approved by the ethics committee

## 3. Clinical Manifestation

Irregular vaginal bleeding, menstrual volume, and vaginal bleeding were manifested.

## 4. Supplementary Examination

Preoperative B-ultrasound examination indicates endometrial thickening and heterogeneous echo. There were reported 2 cases of preoperative diagnostic curettage and 6 cases of hysteroscopy. The preoperative pathological showed the existence of complex atypical hyperplasia of the endometrium, focal carcinogenesis, and endometrioid carcinoma

## 5. Surgical Treatment

They all did single-hole laparoscopic extra fascial total hysterectomy with double adnexal hysterectomy and sentinel lymph node biopsy. Here are the specific steps: make a 2-2.5 cm longitudinal incision in the umbilical cord to cut the skin, rectus abdominis, and peritoneum and after that openly enter the abdominal cavity (see Figure 1). Incision protective cover is used to open the incision (see Figure 2) to connect the upper seal cover (see Figure 3). Then, fill the abdominal cavity with carbon dioxide to form an artificial pneumoperitoneum (pneumoperitoneum pressure is set to 12 mmHg, 1 mmHg = 0.133 kPa). Surgical procedure: Indocyanine green (ICG) is injected into the cervix at 3 and 9 o'clock according to the 2018 NCCN guidelines. ICG powder was diluted to 1.25 mg/ml with 20 ml sterile water before injection. Each site combines shallow (1-3 mm) and deep (1 cm) injections, with a total of 2-4 ml. Then, detection of developed sentinel lymph nodes by OptoMedic fluorescence laparoscopic fluoroscopy (see Figures 4 and 5) is to be excised. Meanwhile, the rapid pathology showed negative results. Therefore, type I extra fascial hysterectomy plus double adnexal hysterectomy was performed routinely, and none of them was converted to laparotomy or porous. The navel suture looked artistical in postoperative (see Figure 6). Operation time is 160.87 ± 40.61, 124-223 min, and blood loss is 68.75 ± 12.31 ml (50-100 ml) in intraoperative. There was no drainage tube that was placed after the operation

## 6. Distribution of SLN

SLN was successfully detected in all 8 cases. The development time of SLN is between 1 and 15 min. The average time is 8 min. There were 32 SLN in total, all of which were developed bilaterally. There were 1 to 3 SLN on each side, and the average number of SLN detected on each side was 2.0. The specific development sites are shown in Table 1

## 7. Postoperative Condition

All 8 cases were treated with flurbiprofen axetil injection 50 mg intravenous drip. It is used for analgesia twice a day for 2 days. Five cases were exhaled within 2 days after the operation, and 3 cases were exhaled on the 3rd day after the operation. The catheter was pulled out routinely 2 days after the operation. Four cases were discharged 3 days after the operation. The rest were required to wait for pathological results, so they were discharged from the hospital for 4 days. The postoperative pathology of the patients is shown in Table 2. All the incisions healed well when we did return visit after one month (see Figure 7). The degree of satisfaction was evaluated, and all of them were very satisfied

## 8. Statistical Method

Statistical analysis used SPSS 20.0 software. The measurement data that obey normal distribution by the normality test are expressed as *x* ± *s*

## 9. Discussion

Endometrial carcinoma is the sixth most common gynecological malignant tumor in the world and it shows a younger trend [1]. The status of lymph node metastasis in patients with endometrial carcinoma is an important index of surgical and pathological staging in the International Federation of Gynecology and Obstetrics (FIGO). Then, we can judge the situation after the expectation to provide a basis for follow-up treatment. Therefore, retroperitoneal lymphadenectomy is required for the staged operation of endometrial carcinoma. However, lymphadenectomy can increase the incidence of related complications, such as lymphedema, lymphocyte, chylous leakage, cellulitis, vascular injury, and nerve injury, which affect the quality of life of the patients [2]. Especially for lymphedema, for some special people who have high requirements for their shape, especially for patients with endometrial cancer with special requirements for the shape of their abdomen and lower limbs, there is no doubt that this kind of traditional operation is a devastating blow to their quality of life and work. Can there be an accurate treatment for early endometrial cancer to reduce complications?

The therapeutic value of retroperitoneal lymphadenectomy for early differentiated endometrial carcinoma is still controversial. The American Gynecological Oncology Group (GOG 33) study showed that the overall risk of pelvic and abdominal para-aortic lymph node metastasis in patients with stage I highly differentiated endometrial cancer was 3% and 2%, respectively. The rate of lymph node metastasis in patients with tumors confined to the endometrium was lower which is about 1% [3]. Another RCT study suggested that there was no difference in PFS and OS in lymph node resection of early endometrial carcinoma system for 5 years [4]. There is no evidence to support that lymphadenectomy can reduce the mortality and recurrence rate of patients or can increase the related complications. Patients with endometrial cancer without high-risk factors can be exempted from lymphadenectomy, but the status of lymph node metastasis needs to be accurately evaluated. At present, the evidence-based medical evidence of SLNB in endometrial cancer recommended by NCCN guidelines is grade 2A, which has high accuracy in predicting lymph node metastasis and has been widely used in the clinic. In 2020, Euscher and Malpica [5] completed a multicenter prospective cohort study, pointing out that SLN has high diagnostic accuracy for endometrial cancer metastasis and can safely replace lymph node dissection. The Professional Committee of Obstetrics and Gynecology of China Research Hospital Association issued an expert consensus on the clinical application of sentinel lymphadenectomy for endometrial cancer in July 2020. It suggested to evaluate the lymph node status of patients with endometrial carcinoma whose lesions are limited to the uterine body before operation and SLNB should be performed first during the operation. Clinically suspected positive lymph nodes should be removed at the same time. And for those patients with failed SLN development should be applied for systematic lymphadenectomy. Secondly, cervical injection of bioactive dye, fluorescent dye, and tracer combined with tracer can be effectively applied to SLNB of endometrial carcinoma. Thirdly, the resected was not only examined pathologically by H&E staining but also carried on the pathological examination of super staging to keep the false negative rate to a minimum for some qualified hospitals. Lastly, it recommends applying SLNB widely for patients with early low-risk endometrial carcinoma for minimally invasive and good tumor safety. It can replace systematic lymphadenectomy.

The development of traditional porous laparoscopy has been relatively mature, and it has been recommended by NCCN guidelines for the early operation of endometrial cancer. However, it will leave four scar marks on their abdomen which also has a certain impact on the types of work that need to expose the abdomen. With the continuous pursuit of beauty and the continuous exploration of new technologies, single-hole laparoscopic surgery came out. It is divided into transumbilical single-hole laparoscopic surgery (laparoendoscopic single-site surgery (LESS)) and endoscopic surgery via natural cavity (natural orifice transluminal endoscopic surgery (NOTES)). LESS is the use of a human natural scar to hide the surgical incision in or around the umbilical hole so that there is almost no scar on the body surface, and even further cosmetic shaping of the navel can be done during the operation. At present, LESS is still in the development stage in gynecology, the operation is mainly benign diseases, and its application in endometrial carcinoma is still being explored. In 2009, Professors Fader and Escobar reported a case of single-hole laparoscopic radical resection of endometrial carcinoma [6]. Mubiao and Huihua [7] performed the first single-hole laparoscopic staging surgery for endometrial cancer in China in 2011. And the results showed that the perioperative result of LESS was similar to that of traditional laparoscopic surgery in the treatment of endometrial cancer. It not only reduced postoperative pain and analgesic requirements but also improved the cosmetic satisfaction of patients. In 2019, Professor Chamber [8] reported that porous laparoscopy, single-hole laparoscopy, and robotic laparoscopy were performed in 150 patients with early endometrial cancer, which is currently the largest multicenter retrospective study. The results are the same as the former, which proves that single-hole laparoscopy is feasible in the surgical treatment of early endometrial carcinoma.

The minimally invasive team of gynecologic tumors in Jiaxing Maternal and Child Health Hospital took the lead in carrying out single-hole laparoscopy combined with menstrual laparoscopy in China. These treatments not only achieve the accurate goal of tumor treatment but also realize the pursuit of beauty for patients with early endometrial cancer who suffer from early endometrial cancer and have special types of work. This also ensures the life and quality of life of the patients to the greatest extent and greatly reduces the difficulty of the operation. However, the author has the following points for attention to this kind of surgery: (1) The best choice for patients is in stage I who without any high-risk factors for endometrial cancer could choose single-hole laparoscopy. However, we recommend patients with high-risk factors could have high-risk abdominal para-aortic lymph node dissection. Otherwise, a single-hole operation will increase the difficulty and risk of the operation and prolong the operation time. Single-hole surgery is not recommended for patients with multiple operations or extreme obesity. Because multiple operations can lead to dense pelvic adhesion and obese patients' intestines affect the visual field and even cause intestinal injury. (2) Cervical injection: It is suggested that intraoperative operation should be performed in more than 20 cases with injection experience to reduce the incidence of false negative. If one side is not developed, it is recommended that this side should make up again to check the image. If there is still not, then we recommend that the negative side of the system be cleaned. As the development time of indocyanine green is 5-10 minutes, cervical injection is recommended after entering the abdomen. (3) Overcome the “chopsticks effect” using the “chopstick technology”; that is, the 10 mm mirror rod is placed in the middle line of the longitudinal axis of the human body, two operating instruments, one left and the other right, are clamped and fixed on one side, and the energy equipment is held on the other side. It is also recommended to use an optical all-in-one mirror; otherwise, the guided beam will affect the operation. (4) Overcome the lack of operational triangles: Beginners suggest the appropriate expansion of umbilical incision to 3 cm. The left- and right-hand instruments need to be long and short. Its tip is relative, and the tail is at a certain distance to form a small operational triangle. Then, the left and right hands cooperate to complete the operation. For the operation of the tip of the operating instrument within the distance of 3 cm, knotting and stitching are generally easier to complete. (5) Treatment of round ligament: Because of the lack of assistant help in single-hole laparoscopic surgery, it is recommended to cut the short round ligament after sentinel lymph node biopsy. It is denied that the surrounding tissue lacks support after amputation of the round ligament, which makes the operation more difficult. (6) Suture of the vaginal stump: Single-hole laparoscopic suture is difficult. It is recommended to use 2-0 inverted thorn sutures, which can reduce the difficulty of sutures and the risk of incision infection. However, it is necessary to inform the family members that the thorn thread is absorbed for a long time and the forbidden lifetime needs to be extended. (7) Postoperative exploration: Due to the tubular visual field and without the assistance of an assistant, single-hole surgery is extremely prone to injury of the urinary catheter and the intestinal canal below the operating hole, so the exploration of the urinary catheter and intestinal tube, especially below the operating hole, is very important after the operation.

This study preliminarily confirmed that LESS combined with sentinel lymph node imaging in the treatment of early endometrial carcinoma in the special population should be safe and feasible, with high aesthetics and satisfaction. However, due to the small number of cases and lack of control, so the next step is we will do a multicenter, double-blind study to get more accurate data to guide the clinic in conjunction with other medical centers.

## Figures and Tables

**Figure 1:** Make a longitudinal incision of 2-2.5 cm in the umbilical region.

**Figure 2:** Incision protective cover to open the incision.

**Figure 3:** Connect the upper seal cover.

**Figure 4:** Developed lymphatic vessels.

**Figure 5:** Development of sentinel lymph nodes during operation (the blue cluster is the sentinel lymph node).

**Figure 6:** Suture of novel incision at the end of the operation.

**Figure 7:** Novel incision appearance one month after the operation.

**Table 1:** Development and distribution of 32 sentinel lymph nodes.

Item	Value
Total check out (*n*)	32
Both sides (*n*(%))	32 (100%)
Sentinel lymph node site (% (number of developing sides/total number of sides))	
Closed hole	37.5 (6/16)
External ilium	43.7 (7/16)
Internal ilium	12.5 (2/16)
Total ilium	6.2 (1/16)

**Table 2:** Postoperative pathological condition about 8 cases of endometrial carcinoma.

Patient serial number	Staging	Pathological type	Degree of differentiation
1	IA	Endometrioid adenocarcinoma	G1
2	IA	Endometrioid adenocarcinoma	G1
3	IA	Endometrioid adenocarcinoma	G2
4	IA	Endometrioid adenocarcinoma	G1
5	IA	Endometrioid adenocarcinoma	G1
6	IA	Atypical hyperplasia of the endometrium	Null
7	IA	Endometrioid adenocarcinoma	G2
8	IA	Atypical hyperplasia of the endometrium	Null

## Data Availability

Please contact corresponding author with reasonable request for the original experimental data and materials.
